# The Effectiveness of Cochlear Implantation for Children of Hereditary Deafness: A Multicenter Retrospective Study

**DOI:** 10.1155/2021/1182949

**Published:** 2021-10-26

**Authors:** Yongzhi Liu, Yelin Li, Yuanyuan Zhao, Liying Ao, Yuting Wen, Haitao Ding

**Affiliations:** ^1^Department of ENT, Inner Mongolia People's Hospital, Hohhot, Inner Mongolia 010021, China; ^2^Department of Clinical Laboratory, Inner Mongolia People's Hospital, Hohhot, Inner Mongolia 010021, China

## Abstract

**Aim:**

To study the effectiveness of cochlear implantation in deaf children with gene mutation.

**Method:**

420 children from three medical centers with cochlear implants were selected. Before wearing the cochlear implant and 6 months after wearing the cochlear implant, the children's rehabilitation efficacy was evaluated through categories of auditory performance (CAP) and speech intelligibility rating (SIR). The SSF-MCDI and MUSS before and after the treatment were also compared.

**Results:**

The CAP and SIR scores of the children after the intervention were higher than those before the intervention (*P* < 0.05). Univariate analysis found that the age of cochlear implantation, parents' education level, and monthly family income were all influencing factors of the CAP score of children with prelingual cochlear implantation (*P* < 0.05). Multivariate logistic regression analysis shows that the age of cochlear implantation <5 years, parents' education level, and monthly household income are all independent risks of CAP scores in children with prelingual deaf cochlear implantation. Univariate analysis found that the age of cochlear implantation, parents' education level, and monthly household income are all based on the SIR scores of children with prelingual cochlear implantation. Multivariate logistic regression analysis can be obtained: the age of cochlear implantation less than 5 years, the education level of parents, and the monthly family income are independent risk factors for SIR scores in children with prelingual deaf cochlear implantation (*P* < 0.05).

**Conclusion:**

The rehabilitation effect of cochlear implants is significant, and the age of cochlear implantation, parents' education level, and monthly family income are all related factors that affect the rehabilitation effect.

## 1. Introduction

Hearing impairment is a common birth defect disease of newborns in clinical practice, and its incidence is about 0.1% to 0.2% [1–3]. There are about 23,000 newborns with different degrees of hearing impairment each year [4]. The vast majority are severe sensorineural hearing loss. Without timely and effective treatment, as the disease progresses, it may pose a serious threat to the normal growth and development of infants and young children and even cause a negative impact on the family and society of the affected child [5, 6]. Hereditary deafness is a common type of deafness. With the popularization and promotion of genetic diagnosis technology, many children with congenital hearing impairment can detect deafness genes. Among cochlear implant patients, the proportion of *GJB2* gene mutations is 26.5% [7].

Cochlear implants, as the only effective method for the treatment of severe or extremely severe sensorineural hearing loss, have been widely used in clinical practice, and more and more children are benefiting from it.

In children diagnosed with GJB2 gene mutation deafness, there were rare studies on the rehabilitation effect of cochlear implantation. Previous studies were limited by their small sample size, retrospective design, and the heterogeneity of included patients. Additionally, previous studies did not systematically study the rehabilitation effect of cochlear implants in terms of auditory and speech intelligibility ability. Therefore, the present study aimed to study for the rehabilitation effect of cochlear implantation for deaf children with gene mutation [8]. We hypothesized that the cochlear implantation could provide rehabilitation effect for children with gene mutation.

## 2. Methods

### 2.1. Study Population

A total of 420 children from 3 medical centers were included in the present study from 2015 to 2019. All of the included children were diagnosed with *GJB2* gene mutation deafness through genetic testing. Inclusion criteria were set as follows: (1) all the included subjects were diagnosed with *GJB2* gene mutation deafness; (2) the patients were younger than 7 years; (3) the cochlear implants worn by the patients were of the same size; and (4) the hearing aids were not improved for 3 to 6 months before the operation. All patients had unilateral cochlear implants. Exclusion criteria: (1) patients with inner ear deformity, facial paralysis, infection, hemorrhage, meningitis, and other related complications; (2) mental and intellectual development abnormalities; and (3) those who withdrew due to various reasons during the study. This study has been approved by the subjects and their families and approved by the hospital ethics committee.

### 2.2. Deafness Genetic Testing

We collected 3 ml of the subject's peripheral blood, used the kit to extract DNA, used a nucleic acid quantifier for concentration and purity testing, and stored the rest at −20°C for later use. We used the “genetic deafness gene chip detection kit” to detect common genetic deafness gene mutation hotspots and analyze the full sequence of related genes in patients with heterozygous mutations.

### 2.3. Data Collection

Baseline data collection: patient's name, gender, contact information, age, parent's education level, dominant hand, implanted ear, and family monthly income. Hearing ability assessment: it is mainly carried out by the categories of auditory performance (CAP). The judgment standards are as follows: if you cannot perceive environmental sounds, it is level 0; if you can perceive environmental sounds but cannot respond, it is level 1, if you can respond to speech sounds, it is level 2; recognizable environmental sounds are level 3; on the basis of not using lip reading, part of the sounds that can be recognized is level 4; on the basis of not using lip reading, common phrases and sentences can be recognized as level 5; on the basis of not using lip reading, the ability to communicate with people is level 6; and the ability to communicate with people on the phone is level 7. Speech proficiency assessment: the speech intelligibility rating (SIR) is used, and the judgment criteria are as follows: coherent language cannot be understood and mainly through sign language communication is level 1; coherent language cannot be understood, but can be carried out through lip reading and language background communication is level 2; continuous language can be understood by the recipients of concentration and lip reading is level 3; continuous language can be understood is level 4 by people without hearing deaf language proficiency; and if continuous language can be understood, the recipient's understanding is level 5. The CAP and SIR scores of children before and after the intervention were compared, and the influencing factors of CAP scores of children with prelingual cochlear implantation and SIR scores of children with prelingual cochlear implantation were analyzed. The vocabulary comprehension ability score and vocabulary expression ability score of the children before and after the intervention were also compared. We used SSF-MCDI and meaningful use of speech scale (MUSS) to evaluate vocabulary comprehension and expression ability.

### 2.4. Statistics

The SPSS 22.0 software was used for statistical processing, the categorical variables were expressed as percentages, and the chi-square test was used. Continuous variables are expressed as mean and standard deviation, using the *t*-test. The influencing factors was evaluated by logistic regression analysis, and the difference was statistically significant with *P* < 0.05.

## 3. Results

### 3.1. Study Population

The baseline characteristics of the patients are shown in Table 1. Among all patients included, there were 215 males and 205 females. The age of the patients ranged from 3 to 7 years, with an average age of 5.12 years. The parents of 290 cases received higher education, and the parents of 130 cases did not receive higher education. There were 208 cases with dominant left hand and 212 cases with dominant right hand. There were 141 patients with cochlear implants on the left side and 279 patients with cochlear implants on the right side. Among all patients with *GJB2* hereditary deafness, 145 cases were 235delC homozygous mutations, 109 cases were 235delC/299_300delAT compound mutations, 235delC/176del16 compound mutations, 35delG/235delC compound mutations, 235delC/512insAACG compound mutations, and 299_300delAT pure, and 235delC mutations were each in 102 cases. There were 35 cases of/427C-T compound mutation, 35delG/299_300delAT compound mutation, and 35delG/605ins46 compound mutation.

### 3.2. Comparison of CAP and SIR Scores of Children before and after Intervention

The average CAP score of patients before treatment intervention was 2.39, and the average CAP score of patients after treatment was 3.56. The average SIR score of patients before treatment intervention was 1.25, and the average SIR score of patients after treatment was 2.38. The CAP and SIR scores of the children after the intervention were higher than those before the intervention (*P* < 0.05). The data are presented in Table 2.

### 3.3. Comparison of SSF-MCDI and MUSS of Children before and after Intervention

The SSF-MCDI before the treatment was 79.1% ± 10.2%, and the MUSS was 81.2% ± 6.8%. After the cochlear implantation, the *SSF-MCDI and MUSS* were improved significantly. The results are presented in Table 3.

### 3.4. Univariate and Multivariate Analysis of CAP Score in Children with a Cochlear Implant

Univariate analysis found that the age of cochlear implantation, the education level of parents, and the monthly family income were all influencing factors of the CAP score of children with cochlear implantation (*P* < 0.05). The child's CAP score was used as the dependent variable, and the age of cochlear implantation, parents' education level, and family monthly income were used as independent variables. Multivariate logistic regression analysis showed that the age of cochlear implantation <5 years, parents' low education level, and low monthly family income were all independent risk factors for the CAP score of children with cochlear implantation (*P* < 0.05). The data are presented in Table 4.

### 3.5. Univariate and Multivariate Analysis of SIR Scores in Children with Cochlear Implantation

Univariate analysis found that the age of cochlear implantation, parents' education level, and monthly family income were all influential factors in the SIR score of children with cochlear implantation (*P* < 0.05). Taking the child's SIR score as the dependent variable and taking cochlear implant age, parents' education level, and family monthly income as independent variables, multivariate logistic regression analysis shows that cochlear implant age <5 years, parents' low level of education, and low monthly household income were independent risk factors for the SIR score of children with prelingual deaf cochlear implantation (*P* < 0.05). The data are presented in Table 5.

## 4. Discussion

Hearing impairment is the most common sensory disability worldwide. Relevant epidemiological data show that the number of hearing disabilities in the world is as high as 360 million, accounting for 5.3% of the global population, including 32 million children [9]. This is the largest number of hearing-impaired children in the world, and the number of hearing-impaired children is increasing by 20,000 to 30,000 every year [10, 11]. Hearing impairment will have a nonnegligible impact on the formation of language, which may cause developmental impairment or stagnation of language function and then affect the psychology, intelligence, and social communication ability of children [12]. Cochlear implantation can create preconditions for the hearing reconstruction of severe or extremely severe children, but there are obvious differences between individuals. Therefore, studying the factors affecting the rehabilitation effect of children with cochlear implantation can provide guidance for improving the rehabilitation effect of children.

The cause of deafness is an important factor that affects the effect of cochlear implantation. Deafness is a common genetic disease in clinical practice [13]. Basically, in 50% of patients, deafness is caused by changes in genetic material. According to different ways of inheritance, inherited deafness can be divided into 5 types: autosomal dominant, autosomal recessive, X-linked inheritance, Y-linked inheritance, and mitochondrial inheritance. Among them, autosomal recessive inherited deafness is the most common, accounting for 75%–80%. Genetic diagnosis of deafness can be used as an effective tool to analyze the etiology of deafness, thereby providing guidance for prevention, treatment, and prognosis [14, 15].

The results of this article showed that the CAP and SIR scores of children after the intervention were higher than those before the intervention (*P* < 0.05). This is highly consistent with previous studies and shows that the rehabilitation effect of cochlear implant patients wearing cochlear implants is significant [16]. Analyzing the reasons, the author believes that the cochlear implant device includes internal and external devices. The main function of the external device is to convert the collected voice signals into electrical signals and then complete the voice coding through a special processing mode and then send them wirelessly to the body for implantation. The latter is to decode the voice signal through the decoding chip after receiving the voice signal, thereby stimulating the patient's auditory nerve and finally producing hearing. Studies have reported that the age of 0–3 is the best period for human speech ability to be acquired, and there is still a chance to acquire strong language ability before the age of 6, and the plasticity of the human brain decreases after the age of 7 until it drops to the age of 12 and then gradually approaching adults. The results of this paper show that age is closely related to the CAP and SIR scores of children with cochlear implants and the CAP and SIR scores of children increase with an increase in age [17]. This suggests that 5–7-year-old children with cochlear implants can obtain better rehabilitation effects.

Studies have confirmed that the earlier a child receives cochlear implantation and the longer he insists on wearing the cochlea after surgery, the better the hearing and speech abilities of the child will be. There are differences in the results of the two studies, and the main reason for this difference may be that the domestic and international common assessment methods have no equivalent effects, so they cannot be directly compared [18]. At the same time, the scores of CAP and SIR mainly depend on the level of central nervous system development, which may make the scores of older children higher than those of younger children. In addition, logistic regression analysis shows that parents' education and monthly family income are closely related to the CAP and SIR scores of children with cochlear implants [19]. The reason is that the author believes that, with the continuous improvement of parents' educational level, the comprehension ability will increase correspondingly, which can actively and effectively cooperate with rehabilitation intervention, thereby better guiding the children to accept the intervention, conducive to the improvement of the children's hearing and speech ability [20]. In addition, the increase of family monthly income can provide favorable conditions for the rehabilitation intervention of children.

In the previous study, Zhou et al. conducted a follow-up evaluation of the effect of auditory rehabilitation on 92 children aged 2 to 7 years after cochlear implant surgery. The results of the study report that the recognition rate of finals at 3, 6, and 12 months were 46%, 73%, and 91%; initial recognition rates were 46%, 66%, and 85% at 3, 6, and 12 months after surgery; the recognition rates of two-syllable words were at 3, 6, and 12 months after surgery [21]. At 12 months, they were 45%, 75%, and 94%. With the increase of postoperative recovery time, the hearing and speech recognition ability of 92 children with artificial cochlear implants has been significantly improved. Domestic scholars have also reported on the postoperative effects of such patients. Liu Jun et al. evaluated 10 children 2 years after the operation. They concluded that patients with GJB2 gene mutations can achieve good rehabilitation results after surgery. This study conducted a one-year longitudinal follow-up evaluation of 42 children [22]. The evaluation results at different stages showed the development rules and trends of the auditory speech recognition ability of such patients and further confirmed that children with GJB2 can obtain good results after cochlear implantation, hearing and speech recognition ability. At the same time, it also provides a basis for the effect of preoperative consultation and rehabilitation for patients with GJB2.

In summary, children with cochlear implants wearing cochlear implants can obtain a relatively ideal rehabilitation effect, and as the age of cochlear implantation increases, the level of education of parents decreases, and the monthly income of the family decreases, and the children will recover. The curative effect has an adverse effect. Therefore, in clinical work, the abovementioned influencing factors can be intervened, which may improve the rehabilitation effect of children which is the purpose of this study.

## Figures and Tables

**Table 1:** The baseline characteristics of the included patients.

The clinical parameters	Patients (*n* = 420, %)

Gender (male)	215 (51.19)
Age	5.12 ± 1.21
Parent's education level (high)	290 (69.04)
Implant ear (left)	141 (33.57)
Monthly family income (high)	15 (3.57)
Dominant hand (left)	208 (49.52)
Duration of severe hearing loss in the implant ear (year)	4.99 ± 1.19
Duration of hearing loss in the nonimplant ear (year)	4.25 ± 2.01
Duration of severe hearing loss in the nonimplant ear (year)	4.12 ± 1.02

**Table 2:** The comparison of CAP and SIR scores of children before and after intervention.

Groups	*N*	CAP	SIR

Before intervention	420	2.39 ± 0.23	1.25 ± 0.19
After intervention	420	3.56 ± 0.15	2.32 ± 0.16
*t*	—	14.24	10.78
*P* value	—	0.001	0.003

**Table 3:** The comparison of SSF-MCDI and MUSS of children before and after intervention.

Groups	*N*	SSF-MCDI	MUSS
Before intervention	420	79.1% ± 10.2%	81.2% ± 6.8%
After intervention	420	89.1% ± 11.2%	91.2% ± 8.9%
*t*	—	12.21	8.92
*P* value	—	0.002	0.001

**Table 4:** Univariate and multivariate analysis of CAP score.

Parameters	Univariate analysis			Multivariate analysis		
	CAP	*t*	*P* value	OR	95% CI	*P* value
*Gender*		0.589	0.557			
Male	3.72 ± 0.66					
Female	3.81 ± 0.69					

*Implant age*		7.636	0.001	1.86	1.05–8.32	0.002
Less than 5	3.14 ± 0.46					
More than 5	4.21 ± 0.73					

*Parents' education level*		4.145	0.001	1.27	1.07–7.21	0.005
Low level	3.37 ± 0.50					
High level	4.01 ± 0.74					

*Dominant hand*		0.406	0.676			
Left	3.74 ± 0.67					
Right	3.80 ± 0.65					

*Implant ear*		0.139	0.890			
Left	3.76 ± 0.62					
Right	3.78 ± 0.67					

*Family income*		9.294	0.001	2.58	0.35–6.28	0.014
Low	3.01 ± 0.48					
High	4.33 ± 0.78					

**Table 5:** Univariate and multivariate analysis of SIR score.

Parameters	Univariate analysis			Multivariate analysis		
	SIR	*t*	*P* value	OR	95% CI	*P* value
*Gender*		0.222	0.825			
Male	2.40 ± 0.81					
Female	2.36 ± 0.77					

*Implant age*		4.303	0.001	1.76	1.06–8.77	0.002
Less than 5	2.01 ± 0.64					
More than 5	2.73 ± 0.82					

*Parents' education level*		4.533	0.001	1.25	1.15–9.22	0.004
Low level	1.96 ± 0.62					
High level	2.77 ± 0.84					

*Dominant hand*		0.114	0.910			
Left	2.37 ± 0.77					
Right	2.39 ± 0.80					

*Implant ear*		0.230	0.819			
Left	2.40 ± 0.82					
Right	2.36 ± 0.73					

*Family income*		5.373	0.001	2.37	1.33–6.29	0.007
Low	1.92 ± 0.60					
High	2.81 ± 0.85					

## Data Availability

The simulation experiment data used to support the findings of this study are available from the corresponding author upon request.
